# Study on the Role and Mechanism of LncRNA ZFasL in Renal Carcinoma

This article has been retracted.

**DOI:** 10.1155/2022/9986549

**Published:** 2022-05-04

**Authors:** Hongbin Shi, Hengyu Zhu, Chao Zhang, Xiaojie Zhou, Wenzhuo Ma, Haoran Xu, Xiaobo Yang

**Affiliations:** ^1^Urology Department, General Hospital of Ningxia Medical University, Yinchuan 750004, Ningxia, China; ^2^Ningxia Medical University, Yinchuan 750004, Ningxia, China

## Abstract

**Background:**

Renal carcinoma is the 7th most common cancer in the world, with the 7th and 6th highest incidence and mortality rates worldwide. Although great progress has been made in the diagnosis and treatment of renal carcinoma, its prognosis is still unsatisfactory. It is important to study the molecular mechanisms of renal carcinoma occurrence and development and to find potential therapeutic targets.

**Objective:**

The main objective is to investigate the effects of long noncoding RNA (lncRNA) ZFAS1 (lncZFAS1) on the proliferation, apoptosis, and migration of renal carcinoma cells and to preliminarily explore its mechanism.

**Methods:**

A qRT-PCR method was used to detect the expression of lncZFAS1 in renal carcinoma tissues and renal carcinoma cells. After shRNA interference with lncZFAS1 expression, the effects of lncZFAS1 on cell proliferation, apoptosis, migration, and invasion were detected by CCK-8 method, flow cytometry, scratch test, and Transwell assay. The effect of the knockdown of lncZFAS1 on the growth of transplanted tumors was examined. The expression of lncZFAS1 in renal carcinoma tissues and renal carcinoma cells was significantly higher than that in paracancerous tissues and normal esophageal epithelial cells. Knockdown of lncZFAS1 significantly inhibited the proliferation, migration, and invasive ability of renal carcinoma cells; upregulated miR-150-5P expression and downregulated HMGA2 expression in renal carcinoma cells; and significantly inhibited the growth of transplanted tumors in nude mice.

**Conclusion:**

Upregulation of miR-150-5P expression was detected after knockdown of lncZFAS1 in renal carcinoma cells, while both mRNA and protein expression levels of HMGA2 were decreased. lncZFAS1 can promote the proliferation and migration of renal carcinoma cells, and the mechanism may be related to the regulation of the miR-150-5P/HMGA2 molecular axis.

## 1. Introduction

The latest global cancer statistics published in 2020 show that renal carcinoma is the 7th most common cancer in the world, with the 7th and 6th highest incidence and mortality rates worldwide, with 572,000 new cases of renal carcinoma and 509,000 deaths worldwide in 2020 [1]. Although great progress has been made in the diagnosis and treatment of renal carcinoma, its prognosis is still unsatisfactory [2]. Therefore, it is important to study the molecular mechanisms of renal carcinoma occurrence and development and to find potential therapeutic targets.

Long-stranded noncoding RNA (lncRNA) is a class of noncoding RNA molecules with transcripts longer than 200 nt, which are widely involved in the regulation of various tumor biological processes, such as cell growth, differentiation, and apoptosis [3, 4]. Recent studies have found that lncZFAS1 (ZNFX1 antisense RNA1) is closely associated with the growth and metastasis of many types of tumors, such as breast cancer [5], gastric cancer [6], nonsmall cell lung cancer [7], bladder cancer [8], and colorectal cancer [9]. lncZFAS1 was initially thought to be a regulator of breast alveolar development and epithelial cell differentiation [10]. Subsequent studies revealed that LncZFAS1 has regulatory functions in a variety of tumors, including lung, liver, and gastric cancers [11]. However, the role and mechanism of lncZFAS1 in renal carcinoma have not been reported in the literature. In this paper, we investigated the possible mechanism of lncZFAS1 expression in renal carcinoma and its effect on the proliferation and migration of renal carcinoma cells. We used the qRT-PCR method to detect the expression of lncZFAS1 in renal carcinoma tissues and renal carcinoma cells. After shRNA interference with lncZFAS1 expression, we used the CCK-8 method, flow cytometry, scratch test, and Transwell assay to detect the effects of lncZFAS1 on cell proliferation, apoptosis, migration, and invasion.

## 2. Materials and Methods

### 2.1. Tissue Samples

Cancer tissue and corresponding paracancerous tissue samples were collected from 32 renal carcinoma patients who did not receive chemotherapy or radiotherapy in our hospital from March 2018 to March 2019 from surgical resection. Patients were aged 42∼73 years, with a mean age of (60.5 ± 5.04) years, 18 males and 14 females. The patients all signed an informed consent form, and the study protocol was approved by the ethics committee of our hospital.

### 2.2. Experimental Animals

SPF class BALB/c nude mice, female, 4 weeks old, 12, weight 16∼20 g, were purchased from Hunan Slaughter Jingda Laboratory Animal Co.

### 2.3. Cells and Viruses

Human normal renal epithelial cell line HK-2 and renal carcinoma cell lines 786-O, ACHN, TK10, A498, 769-P were purchased from the Cell Resource Center of Shanghai Institutes of Biological Sciences, Chinese Academy of Sciences; three shRNA lentiviruses containing specific sh-ZFAS1 against lncZFAS1 and negative control viruses were provided by Guangzhou Ribo Biotechnology Co.

### 2.4. Main Reagents and Instruments

Rabbit anti-human HMGA2 and GAPDH monoclonal antibodies were purchased from Abcam, USA; HRP-labeled sheep anti-rabbit IgG was purchased from Zhengneng Biotechnology Co. Ltd.; transfection reagents were provided by Guangzhou Ribo Biotechnology Co.

### 2.5. Cell Culture and Infection

Human normal esophageal epithelial cell line HK-2 and renal carcinoma cell lines 786-O, ACHN, TK10, A498, 769-P were cultured in 1640 medium containing 10% FBS in a sterile incubator at 37°C with 5% _CO2_ saturation humidity and digested and passaged every 2∼3 d. Three (named No. 1∼3) sh-ZFAS1 lentivirus-infected 786-O and ACHN cells were applied as the silent expression group (lncZFAS1 knockdown group), and negative control virus-infected 786-O and ACHN cells were used as the negative control group.

### 2.6. qRT-PCR Assay

The corresponding tissue samples or groups of cells at the logarithmic growth stage were taken. RNA was extracted according to the RNA extraction kit instructions and quantified. cDNA was synthesized according to the reverse transcription kit instructions. The upstream primer sequence was 5′-CGGGCCTGGACAACTACTA-3′, and the downstream primer sequence was 5′- AAGATGGCTTTCGCACCT-3′. The primers were synthesized by Hunan Dyke Biotechnology Co. The qRT-PCR quantification assay was performed according to the qRT-PCR kit instructions. The number of cycles per well when the fluorescence signal reached the threshold was Ct, and the relative expression level of ZFAS1 was calculated by the ^2−ΔΔCt^ method. The experiment was repeated three times.

### 2.7. Detection of the Effect of Knockdown of lncZFAS1 on the Proliferation of Renal Carcinoma Cells

The CCK-8 method was used. The 786-O and ACHN cells were seeded into 96-well plates at 1 × ^103^ cells/well, and three replicate wells were set up in each group and incubated at 37°C for 24∼96 h. 10 *μ*L of CCK-8 solution was added to each well and incubated at 37°C for 2 h. The absorbance (*A*) value was measured at 450 nm wavelength by an enzyme marker, and the test was repeated three times.

### 2.8. Detection of the Effect of Knockdown of lncZFAS1 on the Migration of Renal Carcinoma Cells Was Performed by Scratch Test

786-O and ACHN cells were inoculated into 6-well plates at ^8 × 105^ cells/well, and 3 replicate wells were set up in each group. The lines were drawn with a 100 *μ*L gun along a straightedge perpendicular to the back of the plate, and the gun should be kept vertical without deflection. After the scribing, wash the plate 2∼3 times with serum-free medium, take microscopic pictures, and measure the width of the scribe at 0 and 48 h. The test was repeated 3 times.

### 2.9. Detection of the Effect of Knockdown of lncZFAS1 on Renal Carcinoma Cell Invasion

Transwell assay was used. 786-O and ACHN cells at the logarithmic growth stage were digested with the trypsin, and the cell concentration was adjusted to 2 × ^106^ cells/mL with serum-free 1640 medium. 50 *μ*L was added to the upper chamber of the Transwell. The chambers were incubated for 24 h at 37°C with 5% CO_2_. The cells were removed from the chambers, the stromal gel and the cells were wiped off with cotton swabs, and the chambers were stained with 0.5% crystal violet solution for 20 min; the residual crystal violet solution was eluted, photographed, and counted, and the test was repeated three times.

### 2.10. Detection of the Effect of Knockdown of lncZFAS1 on Apoptosis of Renal Carcinoma Cells

The Annexin V-FITC/PI assay was used. 786-O and ACHN cells were inoculated into 6-well plates and cultured to logarithmic growth phase, the cell culture medium was collected, resuspended in PBS, and counted, 50,000–100,000 resuspended cells were taken and centrifuged at 200 ×g for 5 min, the supernatant was discarded, 195 *μ*L Annexin V-FITC conjugate was added to resuspend the cells, 5 *μ*L Annexin V-FITC was added, and the cells were incubated at room temperature and protected from light for 10 min. The cells were incubated for 10 min at room temperature and protected from light and centrifuged at 200 ×g for 5 min, the supernatant was discarded, 10 *μ*L of propidium iodide staining solution was added, gently mixed, placed in an ice bath, protected from light, and detected on a flow cytometer, and the test was repeated three times.

### 2.11. Western Blot Analysis Was Performed on 786-O and ACHN Cells at Logarithmic Growth Stage, and Total Protein Was Extracted by Lysis

The analysis conditions were 80 V for 60 min for concentrated gel, 100 V for 90 min for separated gel, semidry membrane transfer, rabbit anti-human HMGA2, and GAPDH monoclonal antibodies as primary antibodies (1 : 200 dilution), HRP-labeled goat anti-rabbit IgG as secondary antibodies (1 : 500 dilution), and ECL luminescent solution development, respectively.

### 2.12. Establishment of a Nude Mouse Transplantation Tumor Model

Twelve nude mice were divided into two groups and inoculated with ACHN cells infected with shRNA lentivirus or negative control virus into the axillae of mice at a rate of 5 × ^106^ cells per mouse. The tumor diameter was measured every 3 d, and the volume (*V*) was calculated according to the following formula. 4 weeks later, the mice were executed, and the tumors were removed for measurement and testing.

(1) $$\begin{array}{c} V={\text{shortest}}^{\text{diameter}2}\times \text{longest diameter}\times 0.5. \end{array}$$

### 2.13. Detection of the Effect of Knockdown of lncZFAS1 on the Growth of Transplanted Tumors in Nude Mice

Immunohistochemical method was used. Tumor tissues were taken, fixed, paraffin-embedded, sectioned, dewaxed, hydrated, antigen repaired, closed, incubated by adding antibodies, DAB color development, dropwise addition of 1% hydrochloric acid alcohol for differentiation, dehydrated, and sealed slices and then observed under the microscope, and images were collected.

### 2.14. Statistical Analysis

The data were analyzed using the statistical software SPSS 19.0. The experimental data were expressed as mean ± standard deviation ($\bar{x}\pm s$), and the mean comparison between groups was analyzed by *t*-test or ANOVA, and the difference was considered statistically significant at *P* < 0.05.

## 3. Results

### 3.1. Expression of lncZFAS1 in Renal Carcinoma Tissues and Cells

qRTPCR results showed that the expression level of lncZFAS1 in cancer tissues was significantly higher than that in paracancerous tissues, and the difference was statistically significant (*t* = 16.09, *P* < 0.000 1), see Figure 1. lncZFAS1 expression in renal carcinoma cell lines 786-O, ACHN, TK10, A498, and 769-P was significantly higher than that in normal esophageal epithelial cell lines, and the differences were all statistically significant (*t* = 15.67, 9.82, 7.37, 5.65, 5.89, respectively, *P* < 0.05). lncZFAS1 was set to have a relative expression of 1 in the normal esophageal epithelial cell line HK-2 and 1 in the renal carcinoma cell lines 786-O, KYSE-510, TK10, A498, and 769-P were 4.80 ± 0.42, 5.14 ± 0.75, 3.58 ± 0.58, 3.19 ± 0.69, and 2.37 ± 0.41, respectively.

### 3.2. The Inhibitory Effect of lncZFAS1 Knockdown on lncZFAS1 Expression in Renal Carcinoma Cells

qRT-PCR results showed that the relative expression levels of lncZFAS1 in both 786-O and ACHN cells with lncZFAS1 knockdown group were significantly lower than those in the negative control group (t 6. 10, 9. 25, 8. 67 and 8. 13, 9. 06, 6. 93, respectively, *p* < 0. 05). 93, all *P* < 0. 05), see Figure 2. Among them, sh-ZFAS1 virus No. 2 was more effective in knocking down lncZFAS1 in both cells and was selected for the follow-up study.

### 3.3. Effect of Knockdown of lncZFAS1 on Proliferation and Apoptosis of Renal Carcinoma Cells

The results of the CCK-8 assay showed that the proliferation ability of 786-O and ACHN cells in the lncZFAS1 knockdown group was significantly reduced compared with the negative control group, and the differences were statistically significant at 48, 72, and 96 h (*t* 4.55, 10.28, 12.01 and 5.17, 8.20, 11.91, *P* < 0.05, respectively), see Figure 3. The results of the Annexin V-FITC/PI assay showed that the proportion of apoptotic cells in both 786-O and ACHN cells in the lncZFAS1 knockdown group was increased compared with the negative control group (*t* 12.51, 10.09, *P* < 0.05), see Figures 4 and 5.

### 3.4. Effect of Knockdown of lncZFAS1 on Migration and Invasion of Renal Carcinoma Cells

The results of the scratch test showed that the migration ability of 786-O and ACHN cells in the lncZFAS1 knockdown group was significantly inhibited compared with the negative control group (*t* 14.31 and 33.70, respectively, *P* < 0.01), see Figures 6 and 7; the results of the Transwell test showed that the invasion ability of 786-O and ACHN cells in the lncZFAS1 knockdown group was significantly inhibited compared with the negative control group (*t* 6.74 and 5.82, respectively, *P* < 0.05), see Figures 6 and 7. Compared with the negative control group, the invasion ability of 786-O and ACHN cells in the lncZFAS1 knockdown group was significantly inhibited (*t* = 6.74, 5.82, *P* < 0.05, respectively), see Figures 8 and 9.

### 3.5. Effect of lncZFAS1 Knockdown on miR-150-5P and HMGA2 Expression in Renal Carcinoma Cells

qRT-PCR results showed that the relative expression levels of miR-150-5P were significantly upregulated in 786-O and ACHN cells in the lncZFAS1 knockdown group compared with the negative control group (both P 0.001), and HMGA2 mRNA relative expression levels were significantly downregulated (P 0.015 and 0.011, respectively), see Figure 10. Western blot analysis showed that HMGA2 protein expression levels were downregulated, see Figures 10 and 11.

### 3.6. Effect of Knockdown of lncZFAS1 on the Growth of Transplanted Tumors in Nude Mice

Compared with the negative control group, the volume of transplanted tumors in the lncZFAS1 knockdown group was significantly reduced (*t* = 6.99, *P* = 0.001), see Figure 12. qRT-PCR results showed that the relative expression level of miR-150-5P in tumor tissues of nude mice in the lncZFAS1 knockdown group was higher than that in the negative control group (*t* = 6.65, *P* = 0.022), see Figure 13. Immunohistochemical results showed that HMGA2 protein expression was inhibited in the tumor tissues of the lncZFAS1 knockdown group of nude mice, see Figure 14.

## 4. Discussion

Renal carcinoma has been in high prevalence in China. Surgery is the main treatment in the early stage because of no obvious or specific clinical symptoms and signs, while radiotherapy is the main treatment in the late stage [12]. Although great progress has been made in the diagnosis and treatment of renal carcinoma, its prognosis is still unsatisfactory [2]. Therefore, it is important to study the molecular mechanisms of renal carcinoma occurrence and development and to find potential therapeutic targets. Long-stranded noncoding RNA (lncRNA) is a class of noncoding RNA molecules with transcripts longer than 200 nt, which are widely involved in the regulation of various tumor biological processes, such as cell growth, differentiation, and apoptosis [3, 4]. Recent studies have found that lncZFAS1 (ZNFX1 antisense RNA1) is closely associated with the growth and metastasis of many types of tumors, such as breast cancer [5], gastric cancer [6], nonsmall cell lung cancer [7], bladder cancer [8], and colorectal cancer [9]. Recent studies have shown that a large number of lncRNAs are abnormally expressed in a variety of tumors and participate in a series of processes such as tumor development as oncogenes or oncogenes suppressors, and lncRNAs may receive widespread attention as therapeutic targets for tumors [11, 13]. It has been reported that miR-150-5P plays an important role in a variety of human diseases, including tumors.

LncZFAS1, located on chromosome 20Q13.13, is an lncRNA transcribed from the antisense chain near the 5' end of protein-coding gene Znfx1, and it has three C/D box snoRNAs (SNORDs): Snord12, Snord12b, and Snord12c [14]. lncZFAS1 was initially thought to be a regulator of breast alveolar development and epithelial cell differentiation [10]. However, the role and mechanism of lncZFAS1 in renal carcinoma have not been reported in the literature. The miR-150-5P can play a biological function in tumor development by regulating its target proteins. In this study, we found that lncZFAS1 was highly expressed in renal carcinoma tissues and cells. Knockdown of lncZFAS1 expression in renal carcinoma cell lines 786-O and ACHN using the shRNA transfection technique revealed that cell proliferation, migration, and invasion were inhibited, while apoptosis was increased, suggesting that lncZFAS1 may play a procancer role in renal carcinoma. Meanwhile, knockdown of lncZFAS1 also inhibited the growth of ACHN cells in nude mice, further confirming the important role of lncZFAS1 in promoting esophageal carcinogenesis and development.

To preliminarily investigate the mechanism by which lncZFAS1 affects the biological function of renal carcinoma cells, this study applied a database to predict miRNAs that may bind to lncZFAS1 and selected the lncZFAS1-miR-150-5P-HMGA2 signaling pathway for validation in conjunction with the report by Zeng et al. [7]. The miR-150-5P can play a biological function in tumor development by regulating its target proteins. For example, miR-150-5P is lowly expressed in glioma and inhibits glioma progression by negatively regulating CTNNB1 and Wnt/*β*-catenin signaling pathways inhibiting glioma progression [15–17]. The miR-150-5P is also low expressed in nonsmall cell lung cancer and inhibits recurrence and metastasis of nonsmall cell lung cancer through negative regulation of HMGA2 and *β*-catenin. HMGA2 is a chromatin-associated protein that is widely involved in a variety of cellular physiological activities, and its major physiological functions include regulation of mitosis and cycle, inducible regulation of gene transcription, induction of transformation, and promotion of cancer cell activation [7, 18].

## 5. Conclusion

In this study, upregulation of miR-150-5P expression was detected after the knockdown of lncZFAS1 in renal carcinoma cells, while both mRNA and protein expression levels of HMGA2 were decreased. This suggests that lncZFAS1 may function by affecting the miR-150-5P/HMGA2 signaling axis, which is consistent with the literature reporting that lncZFAS1 may promote the progression of nonsmall cell lung cancer through miR-150-5P/HMGA2. In summary, the results of this study showed that lncZFAS1 plays a procancer role in renal carcinoma and may serve as a new therapeutic target for renal carcinoma. lncZFAS1 can promote the proliferation and migration of renal carcinoma cells, and the mechanism may be related to the regulation of miR-150-5P/HMGA2 molecular axis.

However, the regulatory role of lncZFAS1 on miR-150-5P and HMGA2 needs to be further validated. This is our future research direction. We need more clinical trials to explore the mechanism of the regulatory role of lncZFAS1 on miR-150-5P and HMGA2.

## Figures and Tables

**Figure 1:** qRT-PCR detection of lncZFAS1 expression in renal carcinoma tissues.

**Figure 2:** qRT-PCR assay of lncZFAS1 expression levels after sh-ZFAS1 virus infection of 786-O (a) and ACHN cells (b). a indicates *P* < 0.05 compared to the negative control group.

**Figure 3:** Detection of the effect of knockdown of lncZFAS1 on the proliferation of 786-O (a) and ACHN cells (b). *a* indicates *P* < 0.05 compared to the negative control group.

**Figure 4:** Flow cytogram of the effect of knockdown of lncZFAS1 on apoptosis in various groups of cells. a, b: 786-O and ACHN cells for the negative control group, respectively; c, d: 786-O and ACHN cells for the lncZFAS1 knockdown group, respectively.

**Figure 5:** Detection of the effect of knockdown of lncZFAS1 on the apoptosis of 786-O and ACHN cells. a indicates *P* < 0.05 compared to the negative control group.

**Figure 6:** Effect of knockdown of ZFAS1 on the migration of renal carcinoma cells detected by scratch test (×200).

**Figure 7:** Effect of knockdown of ZFAS1 on the migration of renal carcinoma cells. aa indicates *P* < 0.01 compared to the negative control group.

**Figure 8:** Transwell assay to detect the effect of knockdown of ZFAS1 on renal carcinoma cell invasion (×200).

**Figure 9:** Effect of knockdown of ZFAS1 on the invasion of renal carcinoma cells. a indicates *P* < 0.05 compared to the negative control group.

**Figure 10:** qRT-PCR detection of the relative expression levels of miR-150-5P (a) and HMGA2 mRNA (b). Compared with negative controls, a indicates *P* < 0.05, and aa indicates *P* < 0.01.

**Figure 11:** Western blot analysis of HMGA2 protein expression levels in renal carcinoma EC10 (a) and ACHN cells (b) after knockdown of lncZFAS1. 1: negative control group; 2: lncZFAS1 knockdown group.

**Figure 12:** Effect of knockdown of lncZFAS1 on the growth of transplanted tumors in nude mice. aa indicates *P* < 0.01 compared to the negative control group. (a) Tumor diameter. (b) Tumor volume.

**Figure 13:** Effect of knockdown of lncZFAS1 on the relative expression level of miR-150-5P in transplanted tumor tissues of nude mice. a indicates *P* < 0.05 compared to the negative control group.

**Figure 14:** Effect of knockdown of lncZFAS1 on HMGA2 protein expression level in transplanted tumor tissues of nude mice (×200). (a) Negative control group; (b) lncZFAS1 knockdown group.

## Data Availability

The datasets used and/or analyzed during the current study are available from the corresponding author on reasonable request.
